# SARS-CoV-2 Induces Expression of Cytokine and MUC5AC/5B in Human Nasal Epithelial Cell through ACE 2 Receptor

**DOI:** 10.1155/2022/2743046

**Published:** 2022-06-02

**Authors:** Sangjae Lee, Hyung Gyun Na, Yoon Seok Choi, Chang Hoon Bae, Si-Youn Song, Yong-Dae Kim

**Affiliations:** ^1^Department of Otorhinolaryngology-Head and Neck Surgery, College of Medicine, Yeungnam University, Daegu, Republic of Korea; ^2^Regional Center for Respiratory Diseases, Yeungnam University Medical Center, Daegu, Republic of Korea

## Abstract

**Background:**

Severe acute respiratory syndrome coronavirus 2 (SARS-CoV-2) causes a novel infectious respiratory disease called COVID-19, which is threatening public health worldwide. SARS-CoV-2 spike proteins connect to the angiotensin converting enzyme 2 (ACE2) receptor through the receptor binding domain and are then activated by the transmembrane protease serine subtype 2 (TMPRSS2). The ACE2 receptor is highly expressed in human nasal epithelial cells. Nasal ciliated cells are primary targets for SARS-CoV-2 replication. However, the effect of SARS-CoV-2 on the upper respiratory tract remains unknown, thus leading to the purpose of our study. We investigate the effects of SARS-CoV-2 on cytokines and mucin expression in human nasal epithelial cells.

**Methods:**

We investigated the effects of the SARS-CoV-2 spike protein receptor binding domain (RBD) on cytokines (IL-1*β*, IL-6, and IL-8) and MUC5AC/5B expression via real-time PCR, ELISA, periodic acid-Schiff (PAS) staining, and immunofluorescence staining in cultured human nasal epithelial cells.

**Results:**

The mRNA expression and protein production of cytokines (IL-1*β*, IL-6, and IL-8) and MUC5AC/5B were increased by SARS-CoV-2 spike protein RBD. ACE2 receptor inhibitor suppressed the expression of cytokines (IL-1*β*, IL-6, and IL-8) and MUC5AC/5B induced by SARS-CoV-2 spike protein RBD.

**Conclusions:**

SARS-CoV-2 induced cytokines (IL-1*β*, IL-6, and IL-8) and MUC5AC/5B expression through the ACE 2 receptor in human nasal epithelial cells. Therefore, ACE2 receptor inhibitors can be an effective therapeutic option for SARS-CoV-2 infection.

## 1. Introduction

New viral respiratory infectious diseases caused by viruses are threatening a global public health since SARS in 2003, followed by MERS in 2012, and coronavirus in 2019. COVID-19, caused by severe acute respiratory syndrome coronavirus 2 (SARS-CoV-2), is a fatal respiratory infectious disease that began to spread in Wuhan, China, in 2019. Recently, several vaccines have been developed and inoculated, but the COVID-19 pandemic is still a worldwide burden.

Airway mucus is essential for the protection of the human respiratory tract. It is known that various mucus genes are expressed in inflammatory respiratory diseases such as COVID-19 [1]. MUC5AC/5B are representative secretory mucin genes related to various inflammatory respiratory diseases and are actively used in research of the respiratory tract [2–5]. Many studies reported that SARS-CoV-2 infection causes changes in various mucus genes and cytokines [1, 6–11]. It is already known that SARS-CoV-2 infection occurs through the renin-angiotensin-aldosterone system (RAAS) and angiotensin converting enzyme 2 (ACE2) receptor serves as the entry of the virus into the human [12–14]. The SARS-CoV-2 spikes connect to the ACE2 receptor through the receptor binding domain (RBD) and are then proteolytically activated by transmembrane protease serine subtype 2 (TMPRSS2) [12–14].

According to recent studies, the expression of ACE2 and TMPRSS2 was noted not only in the respiratory tract but also in the heart, digestive tract, liver, kidney, brain, and other organs affecting the whole body [15]. The expression of ACE2 and TMPRSS2 was low level in airway epithelial cells compared to other organs, but SARS-CoV-2 usually invades through the airway epithelium. In the airway epithelial cells, the expression of ACE2 was the highest in nasal epithelial cells, especially ciliated cells, goblet, and secretory cells [16, 17]. Nasal epithelial cells are pseudostratified columnar epithelial cells, including ciliated and mucus-secreting goblet cells and can serve as the first line of defense in respiratory tract against pathogens like SARS-CoV-2. Also, it is known that nasal ciliated cells are the primary target for SARS-CoV-2 replication in the early stage of COVID-19 among these cells [18]. However, most reports dealing with SARS-CoV-2 are limited to the lower respiratory tract, and the effect of SARS-CoV-2 spike proteins on cytokine and mucin gene expression in the upper respiratory tract has not been reported yet. In addition, studies on the treatment and prevention of SARS-CoV-2 through ACE2 receptor inhibitors are lacking or controversial [19–21].

Therefore, the purpose of this study was to explore the effect of the SARS-CoV-2 spike protein on mucin gene (MUC5AC/5B) and inflammatory cytokines (IL-1*β*, IL-6, and IL-8) expression in human nasal epithelial cells. Also we evaluate the effects of ACE2 receptor inhibitor and dexamethasone on mucin gene (MUC5AC/5B) and inflammatory cytokines (IL-1*β*, IL-6, and IL-8) induced by SARS-CoV-2 spike protein.

## 2. Materials and Methods

### 2.1. Materials

Recombinant SARS-CoV-2 spike protein RBD was acquired from R&D Systems (Minneapolis, MN, USA). ACE2 receptor inhibitor MLN-4760 and dexamethasone were acquired from Sigma-Aldrich (St. Louis, MO, USA). PneumaCult™-Ex Plus Medium and PneumaCult™-ALI Medium were acquired from STEMCELL Technologies (Vancouver, BC, Canada). Primary antibodies were purchased as follows: MUC5AC (ab3649) and MUC5B (ab87376) from Abcam (Cambridge, England, UK), IL-1*β* from Cell Signaling Technology (Danvers, MA, USA), IL-6 from Abcam (Cambridge, England, UK), and IL-8 from Thermo Fisher (Boston, MA, USA). HRP-conjugated secondary antibodies were acquired from Novus Biologicals (Centennial, CO, USA). Goat anti-mouse IgG, IgM (H+L) secondary antibody, Alexa Fluor 488 and goat anti-rabbit IgG (H+L) cross-adsorbed secondary antibody, and Alexa Fluor 546 used for immunofluorescence staining were acquired from Thermo Fisher (Boston, MA, USA). 40,6-Diamidino-2-phenylindole (DAPI) was obtained from Abcam (Cambridge, England, UK).

### 2.2. Air Liquid Interface Culture and Treatment

To obtain human nasal epithelial cells, inferior turbinates were obtained during rhinoplasty surgery in 10 patients who did not have underlying diseases, recent medication history for 4 weeks, family history of allergies, and an allergic reaction on the skin prick test and multisimultaneous allergen tests (MAST). This research was approved by the institutional review board for human studies at the Yeungnam University Medical Center, and the written informed consent was obtained from all 10 patients (IRB No. YUMC 2020-08-029). The harvested epithelial cells were cultured under the air liquid interface. First, the mucosal tissue of the harvested inferior turbinates was cleansed with phosphate buffered saline (PBS) and deposited with dispase (Boehringer Mannheim Biochemica, Mannheim, Germany) in an incubator (37°C, 5% CO_2_, 90 min). The surface of the mucosa was peeled off using a surgical knife and filtered through a mesh after 1% penicillin-streptomycin PBS was added. Epithelial cells were suspended in PneumaCult™-Ex Plus medium and cultured in a 60 mm culture container. Human nasal epithelial cells obtained through this process were cultured in a Transwell system (Corning Incorporated, ME, USA) and PneumaCult™-Ex Plus Medium for 28 days with 95% oxygen and 5% carbon dioxide at a 37°C.

To investigate the effect of the recombinant SARS-CoV-2 spike protein RBD on mucin genes and cytokines, the cells were treated with different concentrations (5 and 10 *μ*g/mL) and cultured for 72 h to induce mucin gene expression and protein production. The control group was cultured in the medium alone for the same time. Additionally, to evaluate the effects of the ACE2 receptor inhibitor and dexamethasone, pretreatment with ACE2 receptor inhibitor MLN-4760 (0.2 and 0.4 nM) or dexamethasone (10 nM) was performed 1 h before the recombinant SARS-CoV-2 spike protein RBD was added.

### 2.3. Real-Time Polymerase Chain Reaction Analysis (Real-Time PCR)

Real-time PCR was conducted using the Gene Amp RNA PCR core kit, iQ SYBR Green Supermix (Bio-Rad, Hercules, CA, USA), the T100TM, and the CFX96 real-time PCR system C1000 Thermal Cyclers (Bio-Rad, Hercules, CA, USA) following the instructions. Primers for IL-1*β*, IL-6, IL-8, MUC5AC (QT01329615, Qiagen, Hilden, Germany), and MUC5B (Bio-Rad 10025636, qHsaCIP0028135, Hercules, CA, USA) were used, and glyceraldehyde-3-phosphate dehydrogenase (GAPDH) was employed as a positive control for each reactions. The primary sequences of the primers used in this experiment are as follows (Table 1). Briefly, the cultured cells were cleansed three times with PBS containing 2% bovine serum albumin, and total cellular RNA was extracted using TRIzol® (Molecular Research Center, Cincinnati, OH, USA). Real-time PCR was performed after synthesizing cDNA by performing reverse transcription PCR. Using iQ SYBR Green Supermix, denaturation (95°C, 15 s) and binding reaction (60°C, 45 s) were repeated 50 times. A melting curve (Roche Applied Science, Mannheim, Germany) was used to evaluate amplification accuracy.

### 2.4. Enzyme-Linked Immunosorbent Assay (ELISA)

The number of MUC5AC/5B and cytokine (IL-1*β*, IL-6, and IL-8) proteins was determined using an enzyme-linked immunosorbent assay (ELISA). Proteins were extracted from the cultured cells using radioimmunoprecipitation assay buffer (Thermo Scientific, Rockford, IL, USA) and quantitatively analyzed using BCA. Twenty micrograms of the extracted proteins was incubated in the F96 Cert. Maxisorp Nunc-Immuno plate (Fisher Scientific, Lenexa, KS, USA) for 24 h at 4°C was then cleansed three times with PBS. After incubating at room temperature for 1 h with 2% bovine serum albumin, the proteins were cleansed with PBS three times to prevent nonspecific binding. And IL-1*β*, IL-6, IL-8, and MUC5AC/5B primary antibodies diluted at a ratio of 1 : 200 were reacted in PBS containing 0.05% Tween 20. After three times cleansing with PBS, HRP-conjugated secondary antibodies diluted at a ratio of 1 : 5,000 in PBS containing 0.05% Tween 20 were added to each well. Each well was cleansed three times with PBS after 1 h. Color development with 3,3′,5,5′-tetramethylbenzidine solution was performed and arrested using 2N-H2SO4. Absorbance was measured using a reader (EL800®, BIO-TEK Instruments, Winooski, VT, USA), and the amount of protein was quantified using a standard curve.

### 2.5. Periodic Acid-Schiff Staining and Immunofluorescence Staining

The cultured cells were fixed in 4% paraformaldehyde for 24 h, dehydrated with stepwise ethanol gradients at 50%, 70%, 80%, 90%, and 100%, treated with xylent, and embedded in paraffin to obtain a 4 *μ*m thick slides. Periodic acid-Schiff (PAS) staining was assessed under a microscope by deparaffinizing the slides and staining them using a PAS staining kit (Sigma-Aldrich, MO, USA). To prevent nonspecific binding, immunofluorescence staining was performed using 5% bovine serum albumin (4°C, 16 h). The primary antibodies for MUC5AC/5B were diluted at a ratio of 1 : 100 with 1% bovine serum albumin, incubated at 4°C for 16 h, and cleansed three times with PBS for 10 min at room temperature. The primary antibodies were incubated with the MUC5AC (Alexa Fluor 488, green) and MUC5B secondary antibodies (Alexa Fluor 546, red) diluted with 1% bovine serum albumin at a ratio of 1 : 200 (2 h, room temperature). The reacted slides were cleansed thrice at room temperature for 10 minutes with PBS and reacted with 4′,6-diamidino-2-phenylindole (DAPI) diluted in PBS at a ratio of 1 : 5000. Staining was assessed using a Nikon fluorescence microscope with 200x magnification (Ti-S, 733551, Nikon, Tokyo, Japan).

### 2.6. Statistics

Statistical analysis was carried out using the SPSS version 22.0 for Windows (IBM Corp., Armonk, NY, USA). All experiments were conducted at least three times, and the means and standard deviations were calculated for sets of measurements. The Mann-Whitney *U* test was used for data comparison. Statistical significance was set at *p* value < 0.05.

## 3. Results

### 3.1. Spike Protein RBD Induced the Expression of ACE2 and TMPRSS2

In the cultured human nasal epithelial cells, spike protein RBD (5 and 10 *μ*g/mL) statistically significantly increased the expression of ACE2 and TMPRSS2 genes (Figure 1) (Table 2).

### 3.2. Spike Protein RBD Induced the Expression of Cytokines

In the cultured human nasal epithelial cells, spike protein RBD (5 and 10 *μ*g/ml) statistically significantly increased the cytokine (IL-1*β*, IL-6, and IL-8) mRNA expression and protein production (Figure 2) (Table 2).

### 3.3. Spike Protein RBD Induced the Expression of MUC5AC/5B

In the cultured human nasal epithelial cells, spike protein RBD (5 and 10 *μ*g/ml) statistically significantly increased the MUC5AC/5B mRNA expression and protein production (Figure 3) (Table 2).

### 3.4. ACE2 Receptor Inhibitor Decreased the Spike Protein RBD-Induced Cytokines

Pretreatment with the ACE2 receptor inhibitor (0.2 and 0.4 nM) statistically significantly inhibited the protein production of cytokines (IL-1*β*, IL-6, and IL-8) increased by the spike protein RBD (Figure 4). As a positive control, dexamethasone (10 nM) presented a similar effect, significantly inhibiting the protein production of cytokines (IL-1*β*, IL-6, and IL-8) increased by spike protein RBD (Figure 4).

### 3.5. ACE2 Receptor Inhibitor Decreased the Spike Protein RBD-Induced MUC5AC/5B

Pretreatment with the ACE2 receptor inhibitor (0.2 and 0.4 nM) statistically significantly inhibited the MUC5AC/5B mRNA expression and protein production increased by spike protein RBD (Figure 5). As a positive control, dexamethasone (10 nM) presented a similar effect, significantly inhibiting the MUC5AC/5B mRNA expression and protein production increased by spike protein RBD (Figure 5). In addition, PAS and immunofluorescence staining confirmed that protein production of MUC5AC/5B was increased by the spike protein RBD and suppressed when ACE2 receptor inhibitor (0.2 and 0.4 nM) or dexamethasone (10 nM) was pretreated (Figure 6).

## 4. Discussions

Cytokines are key factors in the inflammatory reactions of respiratory diseases. Various studies dealing with cytokine changes caused by SARS-CoV-2 have been conducted. In a study by Huang et al., it was shown that COVID-19 patients had higher IL-1*β* and IL-8 levels than normal adults [6]. In a study by Coperchini et al. one of the central factors causing ARDS in COVID-19 patients was found to be an excessive increase of cytokines, the so-called cytokine storm [7]. In a study by Kim et al., cytokine storm was shown to play a key role in the pathogenesis of COVID-19, and medications targeting cytokines are considered a new method of treatment [8]. In our study, the spike protein RBD significantly increased protein production and mRNA expression of inflammatory cytokines (IL-1*β*, IL-6, and IL-8) in the cultured human nasal epithelial cells.

Mucus gene expression is increased by reactive oxygen species, cytokines, and inflammatory mediators of respiratory inflammatory diseases [3–5]. The nature and hypersecretion of the mucus change the course of the disease [22]. In a study by Lu et al., MUC5AC was highly expressed in the lung mucosa of COVID-19 patients [10]. In Yin et al.'s analysis, SARS-CoV-2 infection causes airways to be obstructed by abundant MUC5AC-containg mucus [11]. In our study, the expression of MUC5AC/5B was significantly increased in the cultured human nasal epithelial cells by spike protein RBD.

In previous studies, dexamethasone was reported to reduce not only cytokine production but also the organ damage caused by cytokines in COVID-19 patients [9]. Many studies supporting the effectiveness of systemic steroid treatment in COVID-19 patients have been widely reported, and the WHO recommends dexamethasone treatment in clinical practice [23, 24]. However, since dexamethasone has both anti-inflammatory and proinflammatory effects, its excessive use may lead to an aggravation of the disease by putting patients in an immunosuppressive state [25, 26]. In our study, dexamethasone reduced cytokines and MUC5AC/5B expression induced by SARS-CoV-2 spike RBD protein, providing experimental evidence that supports the clinical results of dexamethasone treatment for COVID-19 patients. However, further research is needed to evaluate the effectiveness and dose adjustment of steroids in COVID-19. Moreover, our study may serve as a basis for laboratory studies on the effect of dexamethasone on COVID-19.

The RAAS system, including ACE2, plays a significant role in COVID-19 infection. There are many studies on SARS-CoV-2 treatment targeting the RAAS system, but the correlation between drugs dealing with RAAS system and their effect on COVID-19 patients is still in debate [21, 27]. ACE2 functions not only as SARS-CoV-2 receptors but also as organ protectors [28]. This two-sided function of ACE2 makes a dilemma in the treatment methods targeting ACE2 [29, 30]. Rodríguez-Puertas explained that the ACE2 receptor promoters are helpful in treating COVID-19 patients [19]. On the contrary, Jia et al. claimed that ACE2 receptor inhibitors can be an option for COVID-19 treatment [20]. In our study, the expression of cytokines and MUC5AC/5B induced by spike protein RBD was significantly decreased by ACE2 receptor inhibitor in the cultured human nasal epithelial cell. Our results may be used as a basis for demonstrating that ACE2 receptor inhibitors may be effective agents in treating COVID-19. Considering the role of ACE2 in protecting organs, if a high dose of ACE2 receptor inhibitors are used systemically, it could inhibit the organ-protective properties of ACE2. To minimize these adverse effects, it would be helpful to use a local ACE2 receptor inhibitors for the nasal mucosa, the first access passage of SARS-CoV-2. In addition, further studies on the treatment of COVID-19 through the combinatorial use of drugs targeting the RAAS system are necessary. In this study, it was confirmed that cytokines and mucin expression induced by the spike protein RBD were reduced by the ACE2 receptor inhibitor. However, when the concentration of the ACE2 receptor inhibitor increased from 0.2 nM to 0.4 nM, the decrease in the expression of cytokines and MUC5AC/5B was not linear. Further laboratory and clinical studies are needed to determine the appropriate concentrations of ACE2 receptor inhibitors to efficiently reduce the expression of cytokines and MUC5AC/5B.

## 5. Conclusions

The expression of inflammatory cytokines (IL-1*β*, IL-6, and IL-8) and MUC5AC/5B was significantly increased by the SARS-CoV-2 spike protein in human nasal epithelial cells. The ACE2 receptor inhibitor decreased the spike protein RBD-induced expression of cytokines and MUC5AC/5B. In conclusion, ACE2 receptor inhibitors may be an efficient option of treatment for SARS-CoV-2.

## Figures and Tables

**Figure 1:** The effects of spike protein RBD on ACE2 and TMPRSS2 expression in the cultured human nasal epithelial cell. Spike protein RBD significantly increased ACE2 mRNA expression in real-time PCR (a). Spike protein RBD significantly increased TMPRSS2 mRNA expression in real-time PCR (b). Three independent experiments were performed. Bars represent the mean ± standard deviation in triplicate. ∗ indicates significance of *p* < 0.05 compared with zero value. Sp. RBD: spike protein receptor binding domain; ACE2: angiotensin converting enzyme 2; TMPRSS2: transmembrane protease serine subtype 2.

**Figure 2:** The effects of spike protein RBD on cytokines expression in the cultured human nasal epithelial cell. Spike protein RBD significantly increased cytokine (IL-1*β*, IL-6, and IL-8) mRNA expression in real-time PCR (a) and protein production in ELISA (b). Three independent experiments were performed. Bars represent the mean ± standard deviation in triplicate ∗ indicates significance of *p* < 0.05 compared with zero value. Sp. RBD: spike protein receptor binding domain: ELISA: enzyme-linked immunosorbent assay.

**Figure 3:** The effects of spike protein RBD on MUC5AC/5B expression in the cultured human nasal epithelial cell. Spike protein RBD significantly increased MUC5AC/5B mRNA expression in real-time PCR (a) and protein production in ELISA (b). Three independent experiments were performed. Bars represent the mean ± standard deviation in triplicate. ∗ indicates significance of *p* < 0.05 compared with zero value. Sp. RBD: spike protein receptor binding domain; ELISA: enzyme-linked immunosorbent assay.

**Figure 4:** The effects of ACE2 receptor inhibitor and dexamethasone on spike protein RBD induced cytokines expression in the cultured human nasal epithelial cell. ACE2 receptor inhibitor and dexamethasone significantly decreased the spike protein RBD-induced IL-1*β* (a), IL-6 (b), and IL-8 (c) protein production in ELISA. Three independent experiments were performed. Bars represent the mean ± standard deviation in triplicate. ∗ indicates significance of *p* < 0.05 compared with zero value. † indicate significance of *p* < 0.05 compared with spike protein RBD (10 *μ*g/ml) only. Sp. RBD: spike protein receptor binding domain; ELISA: enzyme-linked immunosorbent assay; ACE2 I: angiotensin converting enzyme 2 receptor inhibitor; Dexa: dexamethasone.

**Figure 5:** The effects of ACE2 receptor inhibitor and dexamethasone on spike protein RBD induced MUC5AC/5B expression in the cultured human nasal epithelial cell. ACE2 receptor inhibitor and dexamethasone significantly decreased the spike protein RBD-induced MUC5AC/5B m RNA expression in real-time PCR (a and b) and protein production in ELISA (c and d). Three independent experiments were performed. Bars represent the mean ± standard deviation in triplicate. ∗ indicates significance of *p* < 0.05 compared with zero value. † indicate significance of *p* < 0.05 compared with spike protein RBD (10 *μ*g/ml) only. Sp. RBD: spike protein receptor binding domain; ELISA: enzyme-linked immunosorbent assay; ACE2 I: angiotensin converting enzyme 2 receptor inhibitor; Dexa: dexamethasone.

**Figure 6:** The effects of ACE2 receptor inhibitor and dexamethasone on spike protein RBD induced MUC5AC/5B protein production in the cultured human nasal epithelial cell in PAS stain and immunofluorescence staining stain. ACE2 inhibitor and dexamethasone significantly decreased the increasement of MUC5AC (green) and MUC5B (red) protein production in PAS stain and immunofluorescence staining. Sp. RBD: spike protein receptor binding protein; PAS: periodic acid-Schiff staining; ACE2 I: angiotensin converting enzyme 2 receptor inhibitor; Dexa: dexamethasone.

**Table 1:** Primer used for polymerase chain reaction.

Gene	Primary sequence	Annealing temperature (°C)	Product size (bp)
IL-1*β*	F: 5′-ATG CAC CTG TAC GAT CAC TG-3′ R: 5′-ACA AAG GAC ATG GAG AAC ACC-3′	60	142
IL-6	F: 5′-GGT ACA TCC TCG ACG GCA TCT-3′ R: 5′-GTG CCT CTT TGC TGC TTT CAC-3′	60	145
IL-8	F: 5′-ATG ACT TCC AAG CTG GCC GTG GCT-3′ R: 5′-TCT CAG CCC TCT TCA AAA ACT TCT C-3′	60	284
MUC5AC	F: 5′-TCA ACG GAG ACT GCG AGT ACA C-3′ R: 5′-CTT GAT GGC CTT GGA GCA-3′	60	130
MUC5B	F: 5′-CAC ATC CAC CCT TCC AAC-3′ R: 5′-GGC TCA TTG TCG TCT CTG-3′	60	245
GAPDH	F: 5′-CCT CCA AGG AGT AAG ACC CC-3′ R: 5′-AGG GGT CTA CAT GGC AAC TG-3′	60	145

**Table 2:** mRNA gene expression levels (mean ± standard deviation) of the receptors, cytokines, and mucins.

Spike protein Receptor binding domain	Gene						
	ACE2	TMPRSS2	IL-1*β*	IL-6	IL-8	MUC5AC	MUC5B
0 *μ*g/ml	1.000 (0.379)	1.000 (0.229)	1.000 (0.679)	1.000 (0.534)	1.000 (0.309)	1.000 (0.270)	1.000 (0.205)
5 *μ*g/ml	2.146 (0.285)	1.731 (0.422)	3.157 (0.255)	4.471 (0.325)	3.858 (0.410)	2.110 (0.125)	1.566 (0.310)
10 *μ*g/ml	4.518 (0.276)	1.308 (0.397)	7.727 (0.296)	12.810 (0.351)	6.568 (0.527)	2.052 (0.251)	1.764 (0.327)

## Data Availability

The data used to support the findings of this study are included within the article.
